This article has been retracted.

# MicroRNA-335-5p alleviates inflammatory response, airway fibrosis, and autophagy in childhood asthma through targeted regulation of autophagy related 5

**DOI:** 10.1080/21655979.2021.1996315

**Published:** 2022-01-11

**Authors:** Qingbin Liang, Jingjing He, Qian Yang, Qinghua Zhang, Yingjun Xu

**Affiliations:** a Department of Emergency, Qingdao Women and Children’s Hospital, Qingdao City, Shandong Province, China; b Department of Internal Medicine, Qingdao University Staff Hospital, Qingdao City, Shandong Province, China; c Department of Infection, Qingdao Women and Children’s Hospital, Qingdao City, Shandong Province, China; d Department of Pediatrics, Qingdao Women and Children’s Hospital, Qingdao City, Shandong Province, China

**Keywords:** Childhood asthma, MiR-335-5p, ATG5, inflammatory response, airway fibrosis, autophagy

## Abstract

Childhood asthma is the most universal chronic disease, with significant cases reported. Despite the current progress in treatment, prognosis remains poor and the existing drugs cause serious side effects. This investigation explored the mechanisms and use of miR-335-5p on childhood asthma therapy. MiR-335-5p and ATG5 expression was analyzed in clinical plasma samples through RT-qPCR. Airway smooth muscle cells (ASMCs) were cultured, and transfected with miR-335-5p mimic, miR-335-5p inhibitor, and pcDNA3.1-ATG5, or co-transfected with miR-335-5p mimic + pcDNA3.1-ATG5. Asthma cell models were constructed through TGF-β1, and animal models through ovalbumin (OVA). Monocyte-macrophage infiltration in bronchoalveolar lavage fluid (BALF) was determined by May−Grunwald−Giemsa staining, and collagen in lung tissue was assessed via Masson staining. Relationship between miR-335-5p and ATG5 was detected by dual-luciferase assay. Cell proliferation was detected by MTT assay. MiR-335-5p and ATG5 RNA expression was determined by RT-qPCR. Collagen I, collagen III, α-SMA, ATG5, LC3I/II, Beclin-1, and p62 protein expression levels in ASMCs were detected by western blot. MiR-335-5p expression was low, but ATG5 expression was high in childhood asthma. Versus OVA+ mimic NC group, the number of eosinophil and collagen in OVA+ miR-335-5p mimic group were reduced. In contrast to TGF-β1 + mimic NC group, TGF-β1 + miR-335-5p mimic group reduced inflammatory, airway fibrosis, and autophagy in ASMCs. ATG5 was miR-335-5p target. Overexpressing ATG5 significantly reversed the inhibitory effects of miR-335-5p on inflammatory response, fibrosis, and autophagy in ASMCs. Overall, the study concludes that MiR-335-5p alleviate inflammatory response, airway fibrosis, and autophagy in childhood asthma through targeted regulation of ATG5.

## 1. Introduction

Asthma, a chronic inflammatory disease of airways, results in symptoms including recurrent episodes of tachypnea, wheezing, coughing, and chest tightness [1]. Based on the surveys by WTO, there are currently about 235 million people suffering from asthma [2]. Asthma is the most universal chronic disease in children, namely chronic airway inflammation. Bronchial tissue fibrosis is a common pathological feature of childhood asthma [3]. A large number of mitogens in asthmatic lungs, like TGF-β, PDGF, and CTGF, are elevated, which induces airway smooth muscle (ASM) cell proliferation and airway remodeling [4]. Presently, the treatment drugs for asthma include bronchodilators, corticosteroids, leukotriene receptor antagonists, and anti-IgE therapy [5]. However, prognosis is still poor, with potentially serious side effects of chemicals. As a result, the search for new molecular drugs is very vital for targeted therapy of childhood asthma and the improvement of prognosis.

MicroRNAs (miRNAs), short non-coding RNAs, are vital regulators of post-transcriptional regulation of gene expression [6]. Increasing evidences point out that miRNAs act pivotally in asthma pathogenesis, including inflammation and airway remodeling [7-9]. Studies have now revealed that miR-335-5p is down-regulated in childhood asthma miRNA profile [10]. In liver cancer researches, miR-335-5p inhibits liver cancer cell proliferation [11]. In acute coronary syndrome, miR-335-5p reduces atherosclerotic vulnerable plaque formation [8], while in chronic rhinosinusitis, miR-335-5p is inhibits inflammatory response [9]. However, the role of miR-335-5p in childhood asthma and its mechanism are still not clear. According to evidence, miR-335-5p has been confirmed to have a direct binding site with Autophagy related 5 (ATG5) that is among the key proteins to regulate autophagy activity [12]. ATG5 also exerts pathological effects on conditions such as Parkinson [12], and myeloid leukemia [13], through changing autophagy activity. In studies related to osteoporosis, ATG5 silencing reduces proliferation and differentiation of osteoblast proliferation [14]. Studies have found that ATG5 genetic variations, including functional promoter variations, are relative to childhood asthma [15].

The current investigation hypothesized that MicroRNA-335-5p could suppress inflammatory response, airway fibrosis, and autophagy in childhood asthma via a targeted regulation of ATG5. The aim of the research was to determine the expression of miR-355-5p expression in the plasma samples of childhood asthma, to investigate the effects of miR-335-5p on inflammation, fibrosis, and autophagy on ASMC, to assess the association between MiR-335-5p and ATG5 and to determine the effects of ATG5 Overexpressing on miR-335-5p on ASMC inflammatory response, fibrosis, and autophagy.

## 2. Materials and methods

### 2.1. Plasma sample collection

From January 2019 to December 2020, 32 plasma samples were collected from children with asthma and non-asthmatic healthy children in Qingdao Women and Children’s Hospital. Childhood asthma samples were selected in reference to GINA (2021) for children aged 5 years old or more who were diagnosed with asthma [16]. The exclusion criteria: 1. Cases with system immune diseases, diabetes, respiratory malignant tumors or anatomical abnormalities, respiratory foreign bodies, and respiratory tuberculosis; 2. Asthma patients receiving systemic corticosteroids, theophylline, and long-acting β2-agonist/leukotriene receptor antagonist within 4 weeks; 3. Children with severe asthmatic hospitalization; 4. The control group excluding non-asthmatic children with a history of allergies, topic or respiratory diseases [17]. The clinical characteristics of children with asthma and healthy children are shown in Table 1.

**Table 1.** Clinical characteristics of childhood asthma and healthy children

Characteristics	Asthmatic patients	Normal
Number of cases	32	32
Gender (male/female)	15/17	14/18
**Age (years)**	10.88 ± 0.78	10.65 ± 0.93
**Height (cm)**	138.4 ± 4.72	132.7 ± 5.53
**Weight (kg)**	36.5 ± 4.2	42.9 ± 5.1
**pre-FEV1**	92.12 ± 4.75	-
**post-FEV1**	98.95 ± 4.91	-
**pre-FEV1/FVC**	96.5 ± 2.61	-
**post-FEV1/FVC**	99.27 ± 2.08	-
**TLC(103/L)**	7.2 ± 0.45	-
**Hb(g/dL)**	12.1 ± 0.32	-
**Total IgE (IU/mL)**	97.3 ± 24	-
**Medications (corticosteroids/ beta2- agonist/leukotriene receptor antagonist), % of patients**	100%	-

**FEV1: Forced expiratory volume in 1s; FVC: Forced vital capacity; TLC: Total leucocytic count; Hb: Hemoglobin.**

Three mL of blood samples were obtained from each subject via venipuncture, and placed in test tubes containing ethylene diamine tetraacetic acid for centrifugation at 2000 × *g* for 10 minutes at 4°C. Later careful transfer of the plasma was done for the isolation of RNA isolation and their freezing at −20°C for future processing. All the experiments were done after approval from the Ethics Committee of Qingdao Women and Children’s Hospital, as well as from the parents or guardians of all children.

### 2.2. Cell culture

Airway smooth muscle cells (ASMC) were purchased from ATCC. The cells were cultured in Dulbecco’s Modified Eagle Medium (DMEM) (Gibco, US) containing 10% Fetal bovine serum, 100 U/mL penicillin, and 0.1 mg/mL streptomycin. The culture conditions were 37°C and 5% CO_2_, and the cells in logarithmic growth phase were used for the subsequent experiment [18]. The cells in the logarithmic phase were co-transfected with 1, 5, and 10 ng/mL TGF-β1, and cultured for 12, 24, and 48 h, respectively. Cell proliferation was assessed through MTT assay to determine whether the asthma cell model was successfully induced.

### 2.3. Cell transfection

The mimic NC, miR-335-5p mimic, inhibitor NC, miR-335-5p inhibitor (100 nM), pcDNA3.1, and pcDNA3.1-ATG5 (GenePharma, Shanghai, China) were transfected in ASMCs, with 2.5 µg each. The lipofectamine 2000 transfection kit (Thermo Fisher, US) was used for transfection. All transfection experiments were carried out in strict reference to the lipofectamine 2000 transfection instructions. Successfully transfected cells were cultured in DMEM without serum, and later placed incubated for further proliferation [19].

### 2.4. Experimental animals

Twenty-four healthy male BALB/c mice, aged 6–8 weeks, weighing 20–25 g/each, were gained from Hunan SJA Laboratory Animal Co., Ltd. (Changsha, China). All experimental animals were reared in Specific pathogen-free grade sterile laminar flow chamber with alternating light circle for 12 h under constant temperature (22°C–26°C) and constant humidity (55 ± 5%). All animal experiments complied with the Qingdao Women and Children’s Hospital rules and regulations for the management of laboratory animals and the code of operation as well as the associated ethical requirements of laboratory animals.

### 2.5. The induction of asthma model in mice via ovalbumin (OVA)

With six BALB/c mice in each group, except the sham group, 50 μg OVA (200 μL, containing 20 μg OVA and 2 mg aluminum hydroxide, Sigma, US) was intraperitoneally injected into the other three on 1st d and 14th d of the experiment. From the 21st day, 4% OVA solution was atomized and inhaled daily for 30 min for 1 week. Mice in the sham group were treated using the same amount of normal saline instead of OVA atomizer and stimulation solution. Other treatment was the same as the asthma group. In the OVA + miR-335-5p mimic and the OVA+ mimic negative control (NC) groups, intranasal injection of 20 μg miR-335-5p mimic and its NC were conducted once a day 1 h before atomization, and the process was repeated 7 times [20]. Samples were then collected and processed for further experiments.

### 2.6. May−Grunwald−Giemsa staining of BALF samples

BALF samples were mixed slightly and the cell suspensions centrifuged at 300 rpm for 10 min. Pellet was dispensed on the slides. The slides were then stained using the May−Grunwald−Giemsa staining protocol (Differential Quick Staining Kit, Electron Microscopy Sciences, Hatfield, PA, USA), and a coverslip was mounted. A minimum of 400 cells were identified and counted under light microscopy (Olympus BX-46, Tokyo, Japan). Calculation of the mean number of monocyte-macrophage infiltration in each group was done at 200× magnification [21].

### 2.7. Masson staining

Masson staining of mice lung tissues was done as described elsewhere [20]. The accumulation of collagen was determined. The samples were stained with three different staining materials including incubation of tissues with hematoxylin solution, and Ponceau S solution with Acid fuchsin solution, and finally with Phosphomolybdic acid solution. After counter-staining with Aniline blue solution, the images were captured at 200× magnification.

### 2.8. 3-(4,5-Dimethylthiazol-2-yl)-2, 5-diphenyltetrazolium bromide (MTT) assay

Cell viability was determined through MTT assay [22]. After adding 20 µL of MTT solution (5 mg/mL, Sigma) to each well containing the treated ASMCs, the cells were incubated for 3 h and 150 µL Dimethyl Sulfoxide (DMSO) was then added to each well. After promotion of crystal dissolution, absorbance value (OD_490_) was determined using a plate at 490 nm. OD value was set as the ordinate and the time as abscissa to draw MTT curve, and measuring OD value in each group was repeatedly for three times to take the average value.

### 2.9. Reverse transcription quantitative polymerase chain reaction (RT-qPCR)

Total RNA was extracted from plasma and cells using TRIzol Reagent (Life Technologies, NY, USA). The concentration and purity of RNA was determined using ultra-micro spectrophotometer NanoDrop2000 (Thermo Fisher). Reverse transcription on total RNA was carried out using Revert Aid First-Strand cDNA Synthesis Kit (Thermo Fisher). Synthesis of cDNA was done using reverse transcription reaction in PCR amplification machines, and real-time quantitative RT-PCR was eventually done using fluorescent quantitative PCR analyzers (CFX Connect, US). β-actin was as the internal control to standardize RNA expression. U6 served as the internal reference for miRNA. Data analysis was performed via 2^−ΔΔCt^ [23]. The primer sequences and primers of each gene used are shown in Table 2.

**Table 2.** Primer sequences

Name of primer	Sequences
miR-335-5p-F	TGTTTTGAGCGGGGGTCAAGAGC
miR-335-5p-R	CTCTCATTTGCTATATTCA
IL-4-F	AGCAGCTGATCCGATTCCTG
IL-4-R	TGAATGGGTTGACCAAGGGT
IL-13-F	CGAGAAGACCCAGAGGATGC
IL-13-R	GGTGGACACACACCATGGATA
ATG5-F	GCGGTTGAGGCTCAC
ATG5-R	GGATATTCCATGAGT
U6-F	CTCGCTTCGGCAG CACA
U6-R	AACGCTTCACGAATTTGCGT
β-actin-F	CTCCATCCTGGCCTCGCTGT
β-actin-R	GCTGTCACCTTCACCGTTCC

### 2.10. Western blot

Westrern blot assay was performed as previously described elsewhere [24]. Briefly, total proteins quantification was done through the BCA method (Beyotime, Shanghai, China). Subsequently, proteins (30 μg) were separated using 10% sodium dodecyl sulfate-polyacrylamide gel electrophoresis, followed by a transfer into a membrane of polyvinylidene difluoride (PVDF) (Thermo Fisher Scientific). The membrane was later blocked for 1 hour using 5% skimmed milk in TBST, incubated using rabbit anti-human ATG5 (ab109490, 1:1000, Abcam), Beclin-1 (ab210498, 1:1000), LC3I/II (ab192890, 1:1000), p62 (ab109012, 1:1000), collagen I (ab138492, 1:1000), collagen III (ab184993, 1:1000), α-SMA (ab5831, 1:1000), at 4°C overnight. The membrane was subsequently incubated for 1 hr at room temperature using secondary antibody horseradish peroxidase-labeled goat anti-rabbit IgG (1:5000, Solabio). Finally, the band detection was done using the ECL Chemiluminescent Substrate Kit (Thermo Fisher Scientific). β-actin (4970S, 1:1000, Cell Signaling Technology) was as the loading control. Each experiment was performed in triplicate.

### 2.11. Luciferase reporter gene experiment

Dual-luciferase reporter assay was done as previously described [25]. The binding target site of miR-335-5p and ATG5 was predicted using online prediction software Starbase (http://starbase.sysu.edu.cn/)In reference to the prediction findings, design of MUT and WT sequence was for miR-335-5p binding site. There was clone of the sequence fragments and combination with pGL3-promoter vector (Promega) and later transfection of miR-335-5p mimic or its inhibitor or corresponding NC into ASMC cells, respectively. Luciferase Reporter Gene Kit (purchased from Beijing Yuanpinghao Biotechnology Co., Ltd.) was applied to detect fluorescence activity intensity in cells of each group.

### 2.12. Statistical analysis

Data analysis was done using GraphPad prism 8 software. All data were expressed as mean ± standard deviation (SD). Application of T test was for two-group comparisons; one-way analysis of variance (ANOVA) for multiple comparisons among groups; Tukey’s multiple comparisons test was used for subsequent multiple comparisons. Spearman’s rank correlation coefficient was adopted to analyze the correlation between parameters. *P* < 0.05 means statistical significance.

## 3. Results

### 3.1. MiR-335-5p is signally under-expressed in the plasma of children with asthma

Childhood asthma is the most universal chronic disease, with significant cases reported. Despite the current progress in treatment, prognosis remains poor and the existing drugs cause serious side effects. This investigation explored the mechanisms and use of miR-335-5p on childhood asthma therapy. The current investigation hypothesized that MicroRNA-335-5p could suppress inflammatory response, airway fibrosis and autophagy in childhood asthma via a targeted regulation of ATG5.

To ascertain the effects of miR-335-5p on childhood asthma, RT-qPCR was done on a collection of clinical plasma samples. According to the results, miR-335-5p expression was significantly reduced in the plasma samples of the Asthma grouped in comparison to the normal samples (Figure 1(a), *P* < 0.0001). Further RT-qPCR experiments to determine the levels of IL-4 and IL-13 showed a significantly elevated IL-4 and IL-13 levels in Asthma group samples compared to the normal group (Figure 1(b,c), *P* < 0.0001). Based on correlation analysis findings, miR-335-5p was negatively correlated with IL-4 and IL-13 (Figure 1(d,e), *P*< 0.05).

**Figure 1.** MiR-335-5p is apparently under-expressed in children plasma with asthma.

(a) Quantitative PCR to detect miR-335-5p in the plasma of each group; (b) Quantitative PCR to detect IL-4 in the plasma of each group; (c) Quantitative PCR to detect IL-13 in the plasma of each group; (d) Pearson correlation analysis for the relationship between miR-335-5p and IL-4; (e) Pearson correlation analysis for the relationship between miR-335-5p and IL-13. *, *P* < 0.05; ****, *P* < 0.0001. The data represent three separate experiments.

### 3.2. miR-335-5p inhibits ASMC inflammation, fibrosis, and autophagy to relieve asthma

To elucidate the impact of miR-335-5p on childhood asthma, further experiments were done on bronchial smooth muscle cells. MTT assays were done on the experimental cells following treatment of cells under various conditions. According to the results, cells treated with various concentrations of TGF-β1 and various incubation times had a significant increase in their proliferation abilities compared to the controls. The cells treated with 10 ng/mL TGF-β1 and induced for 48 h demonstrated the highest growth (Figure 2(a), *p* < 0.05, *P* < 0.01). As a result, the conditions of 10 ng/mL and 48 h were chosen to construct asthma cell models and named the TGF-β1 group. Relative expression of miR-355-5p was determined in the TGF-b1 treated cells. The observations showed a significantly reduced miR-355-5p expression in the TGF-β1 group compared to the control (Figure 2(b), *p* < 0.01). Therefore, further RT-qPCR experiments confirmed an increased miR-355-5p expression in the TGF-β1 + miR-335-5p mimic as compared to the TGF-β1 and TGF-β1 + mimic NC (Figure 2(c), *p* < 0.01), indicating successfully overexpressing miR-335-5p. In comparison with the TGF-β1 + mimic NC, IL-4 and IL-13 expressions in the TGF-β1 + miR-335-5p mimic were significantly reduced (Figure 2(d,e), *P*< 0.05, *P* < 0.01), indicating that miR-335-5p suppresses ASMC inflammatory response. In contrast to the TGF-β1 + mimic NC, collagen I, collagen III, and α-SMA in the TGF-β1 + miR-335-5p mimic were significantly down-regulated (Figure 2(f), *p* < 0.05, *P* < 0.01), indicating the role of miR-335-5p in the suppression of ASMC fibrosis. In comparison with the TGF-β1 + mimic NC, LC3I/II and Beclin-1 in the TGF-β1 + miR-335-5p mimic were significantly reduced, and p62 was increased (Figure 2(g), *p* < 0.01), indicating that miR-335-5p suppresses autophagy in ASMC. There was no significant difference in the detection indicators between the TGF-β1 and the TGF-β1 + mimic NC. Further exploration of the function of miR-335-5p was done by establishing of a mouse asthma model. Significant elevation of the number of monocyte-macrophage infiltration and collagen was confirmed in the OVA group as compared to the sham (Figure 2(h), I, both *P* < 0.01), whereas the monocyte-macrophage infiltration was significantly reduced the OVA + miR-335-5p mimic in comparison to the OVA + mimic NC (Figure 2(h,i), both *P* < 0.5). Between the OVA and the OVA+ mimic NC was no significant difference of each tested index. In conclusion, miR-335-5p has a certain suppressive effect on asthma.

**Figure 2.** MiR-335-5p represses ASMC inflammatory response, fibrosis and autophagy.

(a) MTT to detect ASMC proliferation ability of each group; (b) Quantitative PCR to detect miR-335-5p in ASMCs of each group; (c) Quantitative PCR to detect miR-335-5p in ASMCs of each group; (d) Quantitative PCR to detect IL-4 in ASMCs of each group; (e) Quantitative PCR to detect IL-13 in ASMCs of each group; (f) Western blot to detect collagen I, collagen III, α-SMA in ASMCs; (g) Western blot to detect LC3I/II, Beclin-1, p62 in ASMCs; (h). The number of eosinophil in the BALF detected by May−Grunwald−Giemsa staining; (i) Masson staining to detect collagen in mouse lung tissue. *, *P* < 0.05; **, *P* < 0.01.

### 3.3. MiR-335-5p regulates asthma through ATG5 targeting

The expression of ATG5 in asthma was determined through RT-qPCR. The results showed that ATG5 was significantly highly expressed in childhood asthma in comparison to the normal group (Figure 3(a), *p* < 0.0001). According to the results of the analysis of correlation, ATG5 was negatively correlated with miR-335-5p (Figure 3(b), *p* < 0.05). To confirm further the relationship between miR-335-5p and ATG5, design of the mutation sites was assessed in ATG5 and miR-335-5p’s 3ʹ-untranslated regions (UTR) (Figure 3(c)), and dual-luciferase reporter gene experiment was conducted. In comparison with the miR-335-5p mimic + WT-ATG5, the miR-335-5p mimic + MT-ATG5 had significantly increased luciferase activity in cells (*P* < 0.01); in contrast to the miR-335-5p inhibitor + WT-ATG5, the luciferase activity in the miR-335-5p inhibitor + MUT-ATG5 was significantly reduced (*P* < 0.01) (Figure 3(d), *p* < 0.01), affirming that miR-335-5p and ATG5 directly bind to each other. After quantitative PCR and western blot experiments, it was found that ATG5 in the miR-335-5p mimic was significantly reduced in comparison to the mimic NC (Figure 3(e,f), *P* < 0.05, *P* < 0.01). In summary, miR-335-5p negatively regulates ATG5 through targeting.

**Figure 3.** MiR-335-5p regulates childhood asthma through ATG5 targeting.

(a) Quantitative PCR to detect ATG5 in the plasma of asthma or normal samples; (b) the Pearson diagram showing the relationship between ATG5 and miR-335-5p. (c) Design of the mutation sites in ATG5 and miR-335-5p 3ʹ-UTR regions; (d) Dual-luciferase reporter gene experiment to calculate the relative luciferase activity of each plasmid; (e) Quantitative PCR to detect ATG5 in ASMCs of each group; (e) Western blot to detect ATG5 in ASMCs of each group. *, *P* < 0.05; **, *P* < 0.01; ****, *P* < 0.0001.

### 3.4. Overexpressing ATG5 reverses the suppressor effect of miR-335-5p on ASMC inflammatory response, fibrosis, and autophagy

To determine the effects of ATG5 overexpression on ASMC, the levels of ATG5 mRNA and protein expressions were determined through RT-qPCR and western blot in TGF-β1, TGF-β1 + mimic NC + pcDNA3.1, TGF-β1 + miR-335-5p-mimic + pcDNA3.1, TGF-β1 + miR-335-5p-mimic + pcDNA3.1 ATG5 cells. The results indicated a reduced ATG5, IL-4 and IL-13 expressions in the TGF-β1 + mimic NC + pcDNA3.1 was significantly reduced in comparison to the TGF-β1 + miR-335-5p-mimic + pcDNA3.1, but elevated in TGF-β1 + miR-335-5p-mimic + pcDNA3.1 in comparison to the TGF-β1 + miR-335-5p-mimic + pcDNA3.1 ATG5 (Figure 4(a-d), all *P* < 0.01), revealing that overexpressing of ATG5 attenuates the inhibitory role of miR-335-5p in ASMC inflammatory response. Collagen I, collagen III, α-SMA, LC3I/II, and Beclin-1 expressions were reduced, while p62 expression was enhanced in the TGF-β1 + mimic NC + pcDNA3.1 in comparison to the TGF-β1 + miR-335-5p-mimic + pcDNA3.1, which was in contrast to the comparison of the TGF-β1 + miR-335-5p-mimic + pcDNA3.1 with the TGF-β1 + miR-335-5p-mimic + pcDNA3.1 ATG5 (Figure 4(e,f), all *P* < 0.01). This observation confirms that overexpressing ATG5 attenuates the suppressive effect of miR-335-5p on ASMC fibrosis and autophagy. In summary, miR-335-5p alleviates childhood asthma inflammatory response, airway fibrosis, and autophagy through targeted regulation of ATG5.

**Figure 4.** Overexpressing of ATG5 reverses the suppressor effects of miR-335-5p on ASMCs inflammatory response, fibrosis and autophagy.

(a) Quantitative PCR to detect ATG5 in ASMCs of each group; (b) Western blot to detect ATG5 in ASMCs of each group; (c) Quantitative PCR to detect IL-4 in ASMCs of each group; (d) Quantitative PCR to detect IL-13 in ASMCs: (e) Western blot to detect collagen I, collagen III, and α-SMA in ASMCs; (f) Western blot to detect LC3I/II, Beclin-1, and p62 in ASMCs. *, *P* < 0.05; **, *P* < 0.01.

## 4. Discussion

Asthmatic attacks usually occur in childhood [26], featuring chronic inflammation and airway remodeling, which seriously threaten children’s health [27]. In the recent years, progress has been made in treating childhood asthma, but there is still a lack of effective strategies [28,29]. Consequently, an urgent need exists to explore new, effective strategies for diagnosing and treating childhood asthma. Studies have revealed that miRNAs result in several chronic respiratory diseases, like childhood asthma [30]. Increasing evidence points out that miRNAs act pivotally in asthma pathogenesis [7]. For example, miR-155 recruits eosinophils and modulates Th2 response to subsequently affect allergic airway inflammation [29]. In this investigation, IL-4 and IL-13 expressions were down-regulated in the presence of miR-355-5p. This is in accordance with various findings of the roles of miRNAs in Th2 differentiation. The miR-355-5p suppressed IL-4 and IL-13 through the down-regulation of B7-H3 type 1 transmembrane protein [31]. MiR-451a restrains airway remodeling through targeting Cadherin 11 in a neonatal mouse allergic asthma model [32].

Studies have revealed that miR-335-5p is suppressed in childhood asthma miRNA profile [10]. In research on periodontitis, miR-335-5p reduces bone loss and inflammation [33]. In sepsis, miR-335-5p also reduces inflammation [34]. Based on clinical sample analysis, miR-335-5p in the plasma samples of children with asthma was visually down-regulated in comparison with healthy children, confirming that miR-335-5p may function positively in childhood asthma. According to the current investigation, miR-355-5p overexpression was observed indicating that miR-335-5p suppressed ASMC inflammatory response, fibrosis, and autophagy. Autophagy acts pivotally in controlling asthma progression [35], and ATG5 is an essential gene for autophagy. Recent research has confirmed that two mutations in ATG5 promoter region are related to childhood asthma [15]. A confirmation was made that ATG5 is a direct target of miR-335-5p. Through overexpressing miR-335-5p, it was found that ATG5 is negatively regulated by miR-335-5p in ASMCs. Further experiments revealed that miR-335-5p exerts biological functions through targeting ATG5. ATG5, an essential autophagosome formation-related protein, modulates various signal pathways like IFN-I, and p53/Rb [36], and is relative to tumorigenesis and inflammation [37]. In asthma studies, there is a positive correlation between ATG5 and various collagen gene expression [38]. The deposition of type I, III, and V collagen as well as of fibronectin is the main reason for fibrosis, which is also the main sign of airway asthma. RhoA/ROCK signaling pathway functions in airway remodeling [39], and in autophagy through active RHOA degradation [40]. Therefore, it was speculated that ATG5 may participate in inflammatory response and airway remodeling in childhood asthma through RhoA/ROCK pathway. Additionally, considering the ceRNA mechanism, it was speculated that lincRNA or circRNA would exist in miR-335-5p upstream to regulate its expression.

The limitation of this study was in deriving the most suitable mice model, of the right age, for childhood asthma. Moreover, it is necessary to investigate time-dependent changes in OVA-induced chronic lung injury. A more detailed analysis of the inflammatory response with regard of ATG5 and miR-335-5p could improve our understanding of how young and adults react to lung injury.

## 5. Conclusion

The results of this investigation confirmed that MicroRNA-335-5p suppress inflammatory response, airway fibrosis, and autophagy in childhood asthma via a targeted regulation of ATG5. Briefly, it was determined that MiR-335-5p is down-regulated in the plasma of asthmatic children, and miR-335-5p inhibits ASMC inflammation, fibrosis, and autophagy to relieve asthma. It was also established that MiR-335-5p regulates childhood asthma through ATG5 targeting. Finally, overexpressing of ATG5 was confirmed to reverse the suppressor effect of miR-335-5p on ASMC inflammatory response, fibrosis, and autophagy. Consequently, miR-355-5p may be used as a potential therapy for asthma in children.
